The article "In Vitro Antibacterial Activity and Mechanism of Vanillic Acid against Carbapenem-Resistant Enterobacter cloacae" was retracted in 2020. Reason: duplicated images.

# In Vitro Antibacterial Activity and Mechanism of Vanillic Acid against Carbapenem-Resistant *Enterobacter cloacae*

**DOI:** 10.3390/antibiotics8040220

**Published:** 2019-11-13

**Authors:** Weidong Qian, Yuting Fu, Miao Liu, Ting Wang, Jianing Zhang, Min Yang, Zhaohuan Sun, Xiang Li, Yongdong Li

**Affiliations:** 1 School of Food and Biological Engineering, Shaanxi University of Science and Technology, Xi’an 710021, China; 201504040401@sust.edu.cn (Y.F.); 1804065@sust.edu.cn (M.L.); Mazedark@foxmail.com (J.Z.); zhaohuansun23@163.com (Z.S.); lixiang@sust.edu.cn (X.L.); 2 Ningbo Municipal Center for Disease Control and Prevention, Ningbo 315010, China; marsliydnb@163.com

**Keywords:** vanillic acid, carbapenem-resistant *Enterobacter cloacae*, cell membrane damage, biofilm, biofilm-associated cells

## Abstract

Vanillic acid (VA) is a flavoring agent found in edible plants and fruits. Few recent studies exhibited robust antibacterial activity of VA against several pathogen microorganisms. However, little was reported about the effect of VA on carbapenem-resistant *Enterobacter cloacae* (CREC). The purpose of the current study was to assess in vitro antimicrobial and antibiofilm activities of VA against CREC. Here, minimum inhibitory concentrations (MIC) of VA against CREC was determined via gradient diffusion method. Furthermore, the antibacterial mode of VA against CREC was elucidated by measuring changes in intracellular adenosine triphosphate (ATP) concentration, intracellular pH (pH_in_), cell membrane potential and membrane integrity. In addition, antibiofilm formation of VA was measured by crystal violet assay and visualized with field emission scanning electron microscopy (FESEM) and confocal laser scanning microscopy (CLSM). The results showed that MIC of VA against *E. cloacae* was 600 μg/mL. VA was capable of inhibiting the growth of CREC and destroying the cell membrane integrity of CREC, as confirmed by the decrease of intracellular ATP concentration, pH_in_ and membrane potential as well as distinctive variation in cellular morphology. Moreover, crystal violet staining, FESEM and CLSM results indicated that VA displayed robust inhibitory effects on biofilm formation of CREC and inactivated biofilm-related CREC cells. These findings revealed that VA exhibits potent antibacterial activity against CREC, and thus has potential to be exploited as a natural preservative to control the CREC associated infections.

## 1. Introduction

*Enterobacter cloacae* (*E. cloacae*) is a common gram-negative, rod-shaped bacterium belonging to the family Enterobacteriaceae and can be frequently detected from human and animal excrement. *E. cloacae* has also been isolated from food processing plants, rice, seafoods and meat products, which can bring out food spoilage [1,2]. Consequently, *E. cloacae* has recently been used as a hygiene indicator in foodstuff processing, and is also one of the most challenging bacterial contaminants of raw and processed meat products, and vegetables [3]. Alarmingly, carbapenem-resistant *E. cloacae* (CREC) that can produce resistance to the last-resort carbapenem antibiotics and compromise these drugs for the treatment of life-threatening infections [4], has been recently detected in seafood originating from Southeast Asia, such as shrimp and clams [5]. This finding indicates that the risk for exposure to CREC extends beyond persons with particular travel histories, previous antimicrobial drug use, or hospitalization, and into the general public.

In addition, another major contributor to food contamination by CREC is the robust nature of the bacterial biofilm. Biofilms can enhance the capacity of the embedded bacteria to survive stresses that are commonly encountered within food processing and act as persistent sources of microbial contamination, thus increasing food safety risks [6]. Therefore, there is an urgent need for expanded availability of ideal preservative agents for CREC in food products.

Vanillic acid (4-hydroxy-3-methoxybenzoic acid, VA), an oxidized form of vanillin, is a phenolic acid derivative found in some forms of vanilla and has been used as preservative, flavoring agent in food, and antioxidant with beneficial biological activities [7]. Previous studies demonstrated that VA possessed antimicrobial activity against foodborne pathogens such as *Staphylococcus aureus*, and *Escherichia coli* [8]. However, there have been no reports on the antimicrobial activity of VA against *E. cloacae* and its mode of action, especially CREC. Thus, the aim of the present study was to determine antimicrobial and antibiofilm activities of VA against CREC.

## 2. Result

### 2.1. Minimum Inhibitory Concentration of VA against CREC

As shown in Table 1, four CREC isolates investigated here manifested carbapenem resistance, as evidenced by MICs of meropenem (MEM) (64 μg/mL), Piperacillin (PIP)/tazobactam (TAZ) (256 μg/mL) and ceftazidime (CAZ) (256 μg/mL). Polymyxin B (0.25 μg/mL) produced inhibitory influence on CREC. Furthermore, the MICs of VA against CREC-3, CREC-7, CREC-16, and CREC-22 were 600 μg/mL. Compared with other isolates, CREC-16 showed higher levels of antibiotic resistance and co-harbored blaKPC and blaNDM-1 genes, and hence was employed for further studies.

### 2.2. Growth Kinetics of CREC Cells in the Presence of VA

The biomass of CREC-16 was decreased when growing in media containing VA at MIC concentration (Figure 1), whereas cells treated with VA at 2MIC presented significantly precipitous loss of viable cell counts, which was below the limit of detection after 24 h. By contrast, at the concentrations of 1/16, 1/8, 1/4, and 1/2MIC, growth curves presented weak increase number and low growth rate. By comparing with different growth curves, higher concentrations of VA led to a sharp decrease in the relative number of living cells compared with lower VA concentrations.

### 2.3. VA Exposure Results in the Decrease in Intracellular Adenosine Triphosphate (ATP)Concentrations, pH and Membrane Potential of CREC

When CREC-16 was exposed to VA at MIC and 2MIC, the intracellular ATP concentration of CREC-16 cells showed a significant decrease (*p* ≤ 0.05) compared to the untreated control group (Figure 2A). Nevertheless, there were no significant differences between cells treated at MIC and 2MIC of VA, but the increase of VA concentration was positively followed by the decrease of ATP levels. Meanwhile, an increase in extracellular ATP of CREC-16 in the concentration-dependent manner was observed, and the action was accompanied by the time-dependent manner (Figure 2B).

Figure 2C showed a significant change in intracellular pH (pH_in)_ of CREC-16 after VA treatment. The original pH_in_ of CREC-16 was 6.41 ± 0.20. The addition of VA at MIC caused a significant (*p* ≤ 0.01) decline in pH_in_ of CREC-16 from 6.41 ± 0.20 to 4.40 ± 0.35. Equivalently, the pH_in_ of CREC-16 cells reduced from 6.41 ± 0.20 to 3.42 ± 0.24 when exposed to VA of 2MIC (*P* ≤ 0.01).

The membrane potential was measured by the intensity of fluorescence. As shown in Figure 2D, the fluorescence intensities of CREC-16 treated with VA at MIC for 2 h were less than those of the untreated control group. Similarly, a significant reduction in membrane potential was found when the concentration of VA increased from MIC to 2MIC (*p* ≤ 0.01).

### 2.4. VA Treatment Improves Cell Membrane Permeability of CREC

Viable cells loaded with cFDA SE exhibit bright green fluorescence, whereas membrane damaged cells stained with PI generate the red fluorescence. As is shown in Figure 3, CREC-16 cells of the untreated control group emitted the green fluorescence (Figure 3A), indicating the physical integrity of cell membrane. Reversely, the cells treated with MIC of VA presented significantly decreased green fluorescence and increased red fluorescence (Figure 3B). With the increase of VA concentration, the green fluorescence intensity diminished, whereas the red fluorescence intensity upraised significantly (Figure 3C).

### 2.5. Changes in Cell Morphology of CREC Occurs in Response to VA

Transmission electron microscopy (TEM) was applied to evaluate the level of cell wall damage and intracellular modification in VA-treated CREC-16. The untreated CREC-16 cells displayed an obvious outline and a peptidoglycan layer (Figure 4A), whereas cells treated with VA at MIC were misshapen, damaged, and disproportionate (Figure 4B). In addition, CREC-16 cells treated with VA at 2MIC exhibited a wavy contour of cytoplasmic membrane, and presented the dense, undifferentiable cellular content, suggesting a significant shrink of cytoplasm (Figure 4C). Hence, VA treatment damaged the cell membrane and cell wall outline of CREC-16.

Field emission scanning electron microscopy (FESEM) images further presented significant changes in cell morphology after treatment with VA. Cells treated with VA at MIC exhibited visibly enlarged and less uniform in size and had a rough surface (Figure 5B) compared with the normal smooth cell surface of the untreated group (Figure 5A). Moreover, cells treated with VA at 2MIC showed substantial surface collapse on cell membrane due to the disruption of cell wall and enlarged (Figure 5C), which presented a positive correlation that was found between the increase in VA concentration and the damage degree of cell membrane.

### 2.6. A Combination of Crystal Violet Staining, FESEM and Confocal Laser Scanning Microscopy Suggests the Inhibitory Effect of VA on Biofilm Formation of CREC

Crystal violet staining method was employed to assess the effect of VA on the inhibition of biofilm growth of CREC-16. As presented in Figure 6, VA exhibited a statistically significant inhibitory effect on the biofilm formation of CREC-16 at various concentrations (*p* ≤ 0.05). The biofilm formation index of the control group was close to 3.6. When treated with 1/32MIC of VA, biofilm formation was inhibited by 45%. More than 95% of the biofilm was inhibited when the concentration of VA was larger than 2MIC.

Besides, according to FESEM and confocal laser scanning microscopy (CLSM) images, a significant inhibition of biofilm formation was observed at MIC and 2MIC VA treatment compared to the untreated group (Figure 7). Moreover, the majority of biofilms was significantly inhibited by VA at 2MIC (Figure 7C,F), indicating that VA exhibits a strong ability to inhibit biofilm formation of CREC-16.

### 2.7. CLSM Images Display the Inactivation of VA against CREC Cells within Biofilms

The inactivation of VA against 36 h-old biofilm-associated CREC-16 cells has been demonstrated in Figure 8. CLSM images of the untreated group appeared almost entirely green (Figure 8A,E), revealing that most of the cell membranes of CREC-16 cells embedded in biofilms were intact and viable. By contrast, CLSM images of CREC-16 cells within biofilm treated with VA at 4MIC appeared numerous bright red, indicating that most of the cell membranes of bacterial cells within biofilms were damaged (Figure 8D,H). However, there were few locations within the biofilm that remained green signal, indicating that a tiny minority of cells within biofilms presented intact and viable in the presence of VA at MIC and 2MIC (Figure 8B,C,F,G). These results indicate that VA can penetrate biofilms by CREC and thus inactivate CREC cells within biofilms. In addition, the heterogeneity of biofilms by CREC makes VA resistant to pass through the thick biofilm enough so that a few biofilm cells of CREC remain still active when exposed to VA.

## 3. Discussion

To our knowledge, this is the first study assessing the antibacterial activity and action mode of VA against CREC. Our results demonstrated the inhibitory effect of VA on cells of CREC-16 and the minimum inhibitory concentration was 600 μg/mL. This is lower than a previous report where, despite the absence of carbapenem resistance, MIC of *Stephania suberosa Forman* extract against *E. cloacae* was 2000 μg/mL [9]. Furthermore, Alves et al. [10] reported that VA with MIC of 1000 μg/mL exhibited excellent activities against *E. coli*, *Pasteurella multocida* and *Neisseria gonorrhoeae*, but the mode of action still remained unexplored. Similarly, growth curves also demonstrated that VA suppressed the growth of CREC-16. These observations demonstrated that VA has a strong antibacterial effect on CREC.

ATP depletion is a common biological alteration that occurs with cellular injury, indicating that ATP could be used as a potential indicator for clarifying the effects of antimicrobial agents on cell membrane integrity. Our results showed that VA-treated CREC-16 presented a remarkable reduction of intracellular ATP, and the alterations of intracellular and extracellular ATP balance in CREC-16 cells were observed, indicating the impairment of cell membrane. These results are consistent with those reported from previous studies. A similar finding that persimmon tannin induced a significant decrease in intracellular ATP concentration of *S. aureus* has been reported by Liu et al. [11]. Shi et al. [12] exhibited that the addition of ferulic acid leads to a significant decline of the intracellular ATP concentration of *Cronobacter sakazakii* cells. Additionally, Kang et al. [13] found that a significant increase in extracellular ATP concentration was observed in *S. aureus* cells treated with peppermint essential oil.

pH_in_ exerts strong influence on cell metabolism, including DNA transcription, protein synthesis, and enzyme activity, and the pH_in_ levels are positively associated with the cell membrane integrity [14]. Hence, the change in pH_in_ could be considered as an indicator of cell membrane integrity. In our study, the change in pH_in_ of CREC-16 was shown to be significantly associated with the VA concentration, where the addition of 2MIC of VA caused the decline of the pH_in_ from 6.41 ± 0.20 to 3.42 ± 0.24. Similarly, Sanchez et al. [15] reported that exposure of *Vibrio cholerae* strains to all extracts tested decreased significantly the pH_in_ from 7.2 to 3.9 ± 0.5 (*P* ≤ 0.05). Gonelimali et al. [14] also displayed that the decrease in pH_in_ was measured in *S. aureus* and *E. coli* cells after exposure to the ethanolic and aqueous extracts of roselle and clove. Therefore, as described in the literatures for plant-derived products, it was concluded that the effect of VA against CREC-16 could be defined as the disruption to the cell membrane integrity. Moreover, hyperpolarization across the cell membrane occurs when VA rush into the cell, thereby making the membrane potential more negative inside, where a significant reduction in membrane potential was observed when the concentration of VA increased from MIC to 2MIC compared with the untreated control group. Similarly, Na et al. [16] reported that the ethanol extract of ginseng reduced the membrane potential of the microbial cells. These results indicated that VA led to plasma membrane hyperpolarization for tested bacteria, which possibly led to irregular cell metabolic activity and cell death.

Our results also demonstrated that CREC-16 cells underwent obvious lysis of the cell envelope by CLSM, as well as the leakage of cytoplasmic components was observed after treatment with VA by TEM. CLSM images exhibited that the permeability of cell membrane enhanced after exposure to VA. The 2MIC-treated CREC-16 cells were almost entirely red, suggesting that the cell membranes were apparently damaged, and substances can move freely in and out of the cell. Meanwhile, FESEM image of CREC-16 cells treated with VA at 2MIC showed that severe morphological alterations appeared in the cell, as well as MIC-treated cells exhibited visibly enlarged and had a rough surface. These changes in physical and morphological of CREC-16 cells have occurred possibly owing to the effect of VA on the permeability and integrity of membrane. In addition, the dense, undifferentiable intracellular materials in VA-treated cells were observed in TEM images. Similarly, CLSM analysis revealed that almost all the bacterial cells were damaged after treatment with VA of 2MIC. Moreover, Matijasevic et al. [17] reported that the morphological changes of *S. aureus* cells exposed to *Coriolus versicolor* methanol extract were observed using FESEM and TEM.

The biofilm has been shown to enhance bacterial resistance to hostile environmental stresses including resistance to antibiotics and antimicrobial agents [18]. Here, our study further exhibited the effects of VA on biofilm formation and inactivation of biofilm-associated cells. The results of crystal violet staining presented that VA at various concentrations exhibited inhibitory effect on the biofilm formation of CREC-16. Meanwhile, FESEM and CLSM images showed that VA-treated cells displayed substantially declined adhesion and survival, suggesting that biofilm formation was significantly inhibited by VA. These results are consistent with a previous observation of Lu et al. [19] that illustrated the inhibitory effects of garlic and *Coptis chinensis* extract on biofilm formation. Besides, CLSM images further showed that VA displayed robust damage effects against biofilm-associated CREC-16 cells. CLSM images of CREC-16 cells within biofilms treated with 4MIC of VA appeared dark red, revealing that most of the cell membranes of cells in biofilms were impaired. Our results were in agreement with the effectiveness of organo-tellurium compound AS101 on the inactivation of *E. cloacae* within biofilms described by Miriam et al. [20].

## 4. Materials and Methods

### 4.1. Reagents

VA (CAS: 121-34-6, HPLC purity ≥ 98%) was obtained from Shanghai Yuanye Biotechnology Co., Ltd. VA was dissolved in dimethyl sulfoxide (DMSO) and filter-sterilized before use. All chemicals and solvents used were of analytical grade.

### 4.2. Bacterial and Culture Condition

Four CREC isolates, originally derived from wound secretions of patients, designated as CREC-3, CREC-7, CREC-16, and CREC-22, were gifted from Dr. Yongdong Li, Ningbo, China. A single colony from the agar plate was inoculated into a test tube containing 3 mL of tryptic soy broth (TSB) medium, and cultured at 37 °C in an incubator overnight with constant shaking at 200 rpm.

### 4.3. Minimum Inhibitory Concentration (MIC) Determination

The MIC was determined according to standard susceptibility broth dilution technique with minor modifications [21]. The culture of CREC was diluted into a 96-well plate (Costar, Corning, NY, USA) using fresh TSB at 10^5^ CFU/mL. Then, the final concentration (0, 200, 400, 600, 800, 1000, 1200, 1400, 1600, 1800, 2000, 2200 μg/mL) of VA and that of polymyxin B (100 μg/mL) were prepared, respectively. After incubation at 37 °C for 24 h, the suspension from each well was inoculated on tryptic soy agar (TSA) plates. MIC was defined as the lowest concentration of VA that totally inhibited visible bacterial growth.

### 4.4. Growth Curves

The growth curves were established according to the method described by Xu et al. [22] with minor modifications to assess the antimicrobial effect of VA against *E. cloacae*. The log-phase bacterial suspension (100 μL, OD_600_ = 0.5) was diluted 100-fold into TSB containing VA at final concentrations of 0, 1/16, 1/8, 1/4, 1/2, 1 and 2 MIC and incubated at 37 °C with gentle shaking of 150 rpm. An aliquot of the culture was removed at different times of growth (0, 2, 4, 6, 8, and 24 h) and plated on tryptic soy agar (TSA) after adequate serial decimal dilutions. Finally, the plates were incubated at 37 °C for 24 h and colonies were counted manually. A kinetic growth or inactivation curve was constructed for each treatment based on the viable cell counts.

### 4.5. Measurement of ATP Levels

The intracellular ATP concentration of CREC was determined based on the method described by Sianglum et al. with some modifications [23]. Exponential-phase CREC at 1 × 10^5^ CFU/mL was treated with 0, 1, and 2 MIC VA at 37 °C for 1, 2 and 3 h, respectively. To assess the amount of intracellular ATP and ATP release, the cells were harvested by centrifugation (8000× *g*, 10 min) and, in parallel, supernatants were filter sterilized and transferred into new tubes to determine extracellular ATP as ATP leakage out of the bacterial cells. Bacterial pellets were washed twice with 10 mM phosphate-buffered saline (PBS, pH 7.0), suspended in the same PBS, and then kept on ice. Intracellular ATP was extracted by DMSO. ATP was measured using the ATP assay kit based on the manual instructions (Beyotime Bioengineering Institute, Shanghai, China). 

### 4.6. Intracellular pH (pH_in_) Measurements

Intracellular pH (pH_in_) was evaluated according to a modified method of Shi et al. [12]. A total of 300 μL of overnight cultures was transferred into 30 mL TSB and incubated at 37 °C for 8 h. Cells were then harvested by centrifugation (8000× *g*, 10 min) and washed twice with 50 mM HEPES (4-(2-hydroxyethyl)-1-piperazineethanesulfonic acid) buffer (pH 8.0) containing 5 mM EDTA, and followed by resuspending the cells in 20 mL of this buffer. Then 3.0 μM of the probe, carboxyfluorescein diacetate succinimidyl ester (cFDA SE, Beyotime Bioengineering Institute, Shanghai, China), was added. The mixture was incubated at 37 °C for 20 min, washed once with 50 mM PBS containing 10 mM MgCl_2_ (pH 7.0), and resuspended in the same buffer. Subsequently, to eliminate nonconjugated cFDA SE, glucose (10 mM, a final concentration) was added and the cells were incubated for an additional 30 min at 37 °C. Finally, cells were washed twice, then resuspended in 50 mM potassium phosphate buffer (pH 7.0), and stored on ice.

An aliquot of cell suspension labeled by fluorescence was treated with VA at three different concentrations (0MIC, MIC and 2MIC), and then transferred into black opaque 96-well flat-bottom plates (Nunc, Copenhagen, Denmark). After exposure for 20 min, the fluorescence intensity was measured under two excitation wavelengths of 440 nm and 490 nm, and the emission wavelength was collected at 520 nm, where excitation and emission slit widths were 9 and 20 nm, respectively. The intracellular pH was determined as the ratio of the fluorescence signal at the pH-sensitive wavelength (490 nm) and that at the pH-insensitive wavelength (440 nm). All measurements were carried out on a microplate reader (Thermo Fisher Scientific, Finland). The system was maintained at 25 °C during the assay. The fluorescence of the cell-free controls was measured and deducted from values for the treated suspension.

Calibration curves were established for cFDA SE loaded cells with buffers of different pH. Buffers consisted of glycine (50 mM), citric acid (50 mM), Na_2_HPO_4_·2H_2_O (50 mM) and KCl (50 mM). The pH was adjusted to various values (2, 3, 4, 5, 6, 7, 8, 9 and 10) with NaOH or HCl. After adjusting pH_in_ and pH_out_ by adding valinomycin (10 μM) and nigrosine (10 μM), the fluorescence intensity was evaluated at 25 °C.

### 4.7. Membrane Potential Assay

Membrane potential was determined according to the method described by Wang et al. with minor modifications [24]. Briefly, the fluorescent probe bis-(1,3-dibutylbarbituric acid) trimethine oxonol [DiBAC_4_(3)] was applied to determine the changes of bacterial membrane potential. Bacteria in the logarithmic phase of growth were harvested by centrifugation at 4000× *g* for 10 min, rinsed twice with 10 mM phosphate-buffered saline (PBS, pH 7.0), and the bacterial concentration was adjusted to 1 × 10^5^ CFU/mL. The bacterial suspensions were treated with VA (0MIC, MIC and 2 MIC) at 37 °C for 2 h and then incubated with DiBAC_4_(3) at 25 °C in the dark for 10 min as well as then washed with PBS. Finally, fluorescence was calculated on a fluorescence microplate reader.

### 4.8. Assessing Bacterial Membrane Integrity

Cell membrane integrity of CREC cells was assessed by confocal laser scanning microscopy (CLSM, Zeiss LSM 880 with Airyscan, Bonn, Germany) according to a modified method of Liu et al. [25]. The mid-logarithmic phase cells were exposed to VA of different concentrations (0MIC, MIC and 2MIC) for 2 h, centrifuged quickly at 8000× *g* for 5 min, and resuspended with equivalent volumes of 0.01 M PBS. After cell suspensions were incubated with the mixture of cFDA SE and propidium iodide (PI) at 37 °C for 15 min, cells were collected and washed with 100 mM PBS to remove excess dyes.

### 4.9. Transmission Electron Microscopy

TEM (G2 F20 S-TWIN, FEI, Hillsboro, USA) observation was performed as described by Joung et al. with some modifications [26]. Exponential-phase CREC cultures were prepared using overnight cultures incubated in TSB at 37 °C until they reached the mid-logarithmic phase of growth. Subsequently, the cell suspension was treated with VA of 0MIC, MIC, 2MIC, and cultured at 37 °C for further 4 h. Then cells were centrifuged (10000× *g*, 8 min) and washed twice with 0.85% NaCl. Following removal of the supernatant, cell pellets were fixed with 2.5% glutaraldehyde at 4 °C for 12 h, and there after dehydrated by 20%, 50%, 70%, 80%, 90% and 100% alcohol for 15 min and finally embedded in resin. Ultrathin samples were cut on ultra-microtome, stained with uranyl acetate, and observed by TEM.

### 4.10. Field Emission Scanning Electron Microscopy

Morphology changes of the bacterial after treatment with VA at different concentrations were observed using a field emission scanning electron microscopy (FESEM, Nova Nano SEM-450, FEI, Eindhoven, Netherlands) according to previous methods [27]. These logarithmic phase cells were allowed to be exposed to VA (0MIC, MIC, 2MIC) at 37 °C for 4 h. Cells were washed with 0.01 M PBS (pH 7.0) and then fixed in 2.5% glutaraldehyde at 4 °C for about 12 h. After treatment, the cells were dehydrated using sequential exposure per ethanol concentrations ranging from 30% to 100% for 10 min. Finally, the cells were fixed on FESEM supports, sputter-coated with gold under vacuum conditions, and cell morphology was examined using FESEM.

### 4.11. Biofilm Examination

The effect of VA on biofilm formation of CREC was tested quantitatively in 96-well plates by modified crystal violet staining assay method as described by Dasagrandhi et al. with some modifications [28]. Following incubation of the CREC cells in the presence of VA at 0, 1/32, 1/16, 1/8, 1/4, 1/2, 1, and 2 MIC for 24 h, planktonic cells and loose adherent cells in the plate were removed with sterile distilled water three times. The cells in the biofilm were then stained with 1% crystal violet (100 µL) and incubated at 28 °C for 15 min and later washed three times with sterile distilled water. The crystal violet bound to the biofilm was then extracted with 30% acetic acid, an aliquot from each well was transferred to a new plate, and the absorbance at 570 nm was determined. Specific biofilm formation index was examined by attaching and stained bacteria (OD_570_) normalized with cell growth (OD_630_).

Effects of VA on the biofilm formation were visually observed by FESEM and CLSM with minor modifications [29]. The slides of cells precultured for 12 h were treated with VA at 0MIC, MIC and 2MIC, and then incubated at 37 °C for 24 h. Subsequently, cells were washed three times with 0.85% NaCl and fixed with 2.5% glutaraldehyde in 200 mM phosphate buffer at 25 °C for 4 h, dehydrated with an ethanol gradient (30%, 60%, 70%, 80%, 90%, and 100%) for 20 min at each concentration. After gold spray treatment, CREC-16 biofilm formation was observed using FESEM, with one point selected for each slide.

In addition, CREC cells grown for 12 h on the slides were precultured and then exposed to VA of different concentrations (0MIC, MIC and 2MIC) for further culture of 24 h. After incubation, the slides of cells were washed three times with 0.85% NaCl. cFDA SE were mixed thoroughly with CREC cells grown well on the slides for direct visual observation of biofilm formation, which were incubated at 25 °C for 15 min. The bacterial biofilm was examined by CLSM, where the fluorescence intensity of cells grown on the slides was measured at excitation/emission wavelengths of 485/542 nm for cFDA SE.

### 4.12. Evaluation of Cell Damages within Biofilms

The damage of CREC cells within biofilm was observed via CLSM according to a previous study [30]. CREC cells grown well for 36 h on the slides were exposed to VA (0MIC, MIC, 2MIC and 4MIC) at 37 °C for 4 h, then washed three times and resuspended with 0.85% NaCl. Then, a combination of fluorescent dyes of cFDA SE and PI was mixed thoroughly with 36-h-old biofilm CREC cells, and the mixture was further incubated at 25 °C for 15 min. Finally, the cell damage was examined by CLSM.

### 4.13. Statistical Analysis

All experiments were performed independently three times, and each biological replicate included two technical replicates. Results were analyzed utilizing using Origin 8.5 Statistics. All data were expressed as mean values and standard deviation (SD). Differences are considered significant at *p* ≤ 0.01.

## 5. Conclusions

In summary, VA was effective in inactivating both CREC cells and biofilm formation. VA could induce in cell lysis resulting in the cell membrane damage and leakage of intracellular components of CREC cells. Additionally, VA at 2MIC can inactivate biofilm CREC cells, and thus has potential use as natural antibacterial agents to control CREC contamination in the food industry.

## Figures and Tables

**Figure 1:** Effect of VA on the growth of CREC-16. Bacterial cells were grown in TSB with 0, 1/16, 1/8, 1/4, 1/2, 1 and 2MIC of VA at 37 °C. The error bars represent standard deviation of three replicates.

**Figure 2:** Effects of VA on intracellular (**A**) and extracellular (**B**) ATP levels, intracellular pH (pH_in_) (**C**) and membrane potential (**D**) of CREC-16. Values represent the mean of triplicate measurements. Bars represent the standard deviation (n = 3). * *p* < 0.05, ** *p* < 0.01.

**Figure 3:** Effects of VA on cell membrane integrity of CREC-16 by confocal laser scanning microscopy. (**A**) CREC-16 cells treated with 1% DMSO; (**B**) CREC-16 cells treated with VA at MIC; (**C**) CREC-16 cells treated with VA at 2MIC.

**Figure 4:** Effects of VA on cell structure of CREC-16 by transmission electron microscopy. (**A**) CREC-16 cells exposed to 1% DMSO; (**B**) CREC-16 cells exposed to VA at MIC; (**C**) CREC-16 cells exposed to VA at 2MIC.

**Figure 5:** Effects of VA on cell morphology of CREC-16 by field emission scanning electron microscopy. (**A**) CREC-16 cells treated with 1% DMSO; (**B**) CREC-16 cells treated with VA at MIC; (**C**) CREC-16 cells treated with VA at 2MIC (magnification of 100,000×).

**Figure 6:** Effects of VA on biofilm formation of CREC-16. Biofilm formation index was determined in the presence of VA at various concentrations in 96-well plates via crystal violet staining.

**Figure 7:** Effects of VA on biofilm formation of CREC-16. Photographs of FESEM (**A**–**C**, magnification of 10,000×) and CLSM (**D**–**F**, three-dimension). (**A**,**D**) CREC-16 cells treated with 1% DMSO; (**B**,**E**) CREC-16 cells treated with VA at MIC; (**C**,**F**): CREC-16 cells treated with VA at 2MIC.

**Figure 8:** Inactivation of VA against CREC-16 cells within biofilms. Plane (**A**–**D**) and three-dimensional (**E**–**H**) images of CLSM. (**A**,**E**) CREC-16 cells within biofilms untreated with VA; (**B**,**F**) CREC-16 cells within biofilms treated with VA at MIC; (**C**,**G**) CREC-16 cells within biofilms treated with VA at 2MIC; (**D**,**H**) CREC-16 cells within biofilms treated with VA at 4MIC.

**Table 1:** Minimum inhibitory concentration of vanillic acid and antibiotics against four carbapenem-resistant *Enterobacter cloacae* strains.

Strain	Carbapenemase Genes	MIC (μg/mL)						
		VA	IMP	MEM	PIP/TAZ	CTX	CAZ	Polymyxin B
CREC-3	NDM-1	600	32	32	>256	>256	>128	0.25
CREC-7	IMP	600	16	32	>128	>256	>128	0.25
CREC-16	KPC, NDM-1	600	32	64	>256	>256	>256	0.25
CREC-22	KPC	600	16	64	>256	>256	>128	0.25

Note: NDM-1, New Delhi metallo-β-lactamase-1; IMP, imipenemase metallo-β-lactamase; KPC, *Klebsiella pneumoniae* carbapenemase.
